# Dysregulation of Circadian Clock Genes Associated with Tumor Immunity and Prognosis in Patients with Colon Cancer

**DOI:** 10.1155/2022/4957996

**Published:** 2022-07-16

**Authors:** Yongshan He, Yuanyuan Chen, Xuan Dai, Shiyong Huang

**Affiliations:** Department of Colorectal Surgery, School of Medicine, Xinhua Hospital Affiliated to Shanghai Jiao Tong University, No. 1665 Kongjiang Road, Shanghai 200092, China

## Abstract

Early research shows that disrupting the circadian rhythm increases the risk of various cancers. However, the roles of circadian clock genes in colorectal cancer, which is becoming more common and lethal in China, remained to be unclear. In conclusion, the present study has demonstrated that multiple CCGs were dysregulated and frequently mutated in CRC samples by analyzing the TCGA database. The higher expression levels of REV1, ADCYAP1, CSNK1D, NR1D1, CSNK1E, and CRY2 had a strong link with shorter DFS time in CRC patients, demonstrating that CCGs had an important regulatory role in CRC development. Moreover, 513 CRC tumor samples were divided into 3 categories, namely, cluster1 (*n* = 428), cluster2 (*n* = 83), and cluster 3 (*n* = 109), based on the expression levels of the CCGs. Clinical significance analysis showed that the overall survival and disease-free survival of cluster 2 and cluster 3 were significantly shorter than those of cluster 1. The stemness scores in cluster 1 and cluster 2 were significantly higher than those of cluster 3 CRC samples. Clinically, we found that the C3 subtype had significantly higher percentage of T3/T4, N1/N2, and grades III and IV than groups C1 or C2. In addition, we reported that different CRC clusters had significantly different tumor-infiltrating immune cell signatures. Finally, pancancer analysis showed that higher expression of CSNK1D was correlated with shorter DFS time in multiple cancer types, such as COAD and LIHC, and was dysregulated in various cancers. In conclusion, we effectively developed a CCG-related predictive model and opened up new avenues for research into immune regulatory mechanisms and the development of immunotherapy for CRC.

## 1. Introduction

Circadian rhythms are required for several biological activities, including metabolism, regeneration, immunology, and endocrinology [1]. Circadian rhythms regulate all human tissues through incredibly intricate mechanisms [2]. The molecular clock is comprised of a core clock gene loop. Circadian rhythm-controlled genes have key roles in tumor processes such as DNA damage and repair, apoptosis, cell proliferation, and metastasis [3]. A growing number of studies have sought to investigate the association between circadian rhythms and cancer in recent years [4, 5]. Early research shows that disrupting the circadian rhythm increases the risk of various cancers, including lung, prostate, breast, colon, endometrial, liver, pancreatic, and kidney cancers [6]. For instance, BMAL1 is vital in the prevention of breast cancer [7]. PER2 overexpression accelerates the growth of oral squamous cell carcinoma [8], and overexpression of NR1D1 may contribute to the development of kidney cell carcinoma [9]. In the pan renal cell carcinoma, circadian clock genes (CCGs) govern immunity, the cell cycle, and apoptosis [9]. Furthermore, persistent jet lag-induced gene deregulation and liver metabolic inefficiency can enhance hepatocarcinogenesis [10]. Nine circadian clock genes, including CCSNK1E, DBP, and NR1D2, were discovered as major prognostic markers in prostate cancer and were utilized to build a risk score model based on them [11]. Previous research has also demonstrated that disturbance of normal rhythms and malfunction of CCGs contribute to the formation and progression of various cancer types, as well as affect the tumor immune cycle function [12]. Previous research has indicated that cancer chronotherapy or scheduled chemotherapy delivery based on circadian rhythm may lessen drug toxicity [13]. Several animal model-based investigations have found that medicines targeting circadian rhythm genes, such as ROR synthesis agonists, can increase anticancer immunity activation [14]. The significance of the circadian clock in prognostic evaluation and its clinical consequences in COAD, on the other hand, are rarely studied. According to one study, CLOCK, CRY1, and NR1D1 mRNA expression was raised in COAD tissue. A bioinformatic study revealed that circadian rhythm genes were mostly associated with the glucocorticoid receptor pathway [15]. However, the functions of CCGs in the colorectal cancer remained largely to be unclear.

Colorectal cancer is becoming more common and lethal in China, with 0.37 million new cases and 0.19 million deaths, respectively [16, 17]. The incidence of colon cancer has considerably grown, and the majority of patients are detected in the middle or late stages [16, 17]. As a result, detecting CRC is a critical duty at the moment. Previous research has demonstrated that full loss of p53 expression indicates a poor outcome in CRC [18]. TMED3 expression has been linked to a poor outcome in CRC [19]. Numerous research has been conducted to study the association between microsatellite instability (MSI) and the prognosis of CRC. The prognosis of CRC with MSI is much better than that of CRC with intact mismatch repair [20].

Immunotherapy has shown great progression in eliminating malignant cells by using the innate processes of the host immune system throughout the last decade, transforming the treatment landscape of many malignancies [21]. Immune checkpoint inhibition (ICI) has proven substantial effectiveness in cancer treatment techniques. ICI significantly increases overall survival (OS) time in patients with melanoma and lung cancer [21]. ICI stimulates the adaptive immune system to prevent immune escape caused by the activation of immune checkpoint cascades such as PD-1 or PD-L1 or CTLA-4 [22]. PD-1 is found on activated lymphocyte cells, which bind to PD-L1 expressed on tumor cells [22]. When activated, the PD-1/PD-L1 axis generates inhibitory signals, resulting in T cell depletion and inactivation [22]. The FDA-approved PD-1 inhibitors pembrolizumab for the treatment of dMMR/MSI-H CRC [23]. Recently, the FDA has also authorized ipilimumab, a CTLA-4 antibody, in conjunction with nivolumab in patients with CRC. Although PD-L1 is the most important prognostic biomarker for immunotherapy, PD-L1 expression was not related to better OS in the pembrolizumab phase II study in MSI-H CRC [24]. As a result, new biomarkers for predicting immunotherapy effectiveness are required.

## 2. Materials and Methods

### 2.1. Datasets and Preprocessing

The TCGA database was utilized to acquire CRC data. The TCGA database included 620 CRC tissues. RNA sequence data and clinicopathological characteristics were analyzed. R software was used for all subsequent statistical studies. *P* < 0.05 was used as the screening criterion for the differential expression of CCGs.

### 2.2. Characterization of Molecular Subtypes of CRC

The gene list of the core circadian clock genes was downloaded from The Molecular Signatures Database (MSigDB) [25, 26]. We aimed to see whether the expression profile of CCGs may help us differentiate between CRC subtypes. 29 CCGs were selected for further ConsensusClusterPlus analysis. The Euclidean distance metric was used to calculate the similarity distance between samples. The samples were clustered over 1000 iterations using the k-means clustering technique. The number of clusters ranged from 2 to 8, and the best partition was chosen by assessing the consensus cumulative distribution function (CDF). The PCA was performed using the R package for R v3.6.0.

### 2.3. Immune Signature Analysis in CRC Molecular Subtypes

The CIBERSORT method [27] was used to calculate the expression scores of microenvironmental variables (tumor, immunological, and stromal purity). TIMER was used to examine the correlation between tumor samples and six tumor-infiltrating cells [28]. The immunological signature and checkpoint gene expression levels were also examined in all molecular subtypes. The analysis of variance (ANOVA) test was used to examine different CRC subtypes. Bonferroni correction was used for multiple testing.

### 2.4. Establishment of Prognostic Signature

CRC data from 620 patients from the TCGA database was retrieved for the identification of prognosis-related CCGs. We constructed a prediction signature for the CCGs stratified by the risk score using a univariate Cox proportional regression analysis and the least-absolute shrinkage and selection operator (Lasso) regression (risk score = EXP CCGs *n* coefficient*n* + EXP CCGs 1 coefficient1 + EXP CCGs 2 coefficient2 + ⋯+EXP CCGs *n* coefficient*n*). The risk score for each CRC patient was then computed. Based on the median risk score, the CRC patient was categorized as risk score-high or low group. The ROC curves were computed using the “survivalROC” program to evaluate the specificity and sensitivity of the prognosis model.

### 2.5. Analysis of mRNAsi Levels and MSI Levels

The mRNAsi was calculated using the OCLR machine-learning algorithm [29]. MSI analysis with MANTIS was performed as previously described [30].

### 2.6. Statistical Methods

To evaluate the connection between molecular subtypes and clinical factors, Fisher's exact test or the chi-square test was utilized. These statistics were generated using the R software and were two sided.

## 3. Results

### 3.1. The Expression and Genetic Variation Profile of CCGs in CRC

To begin with, we discovered that ARNTL2, CSNK1E, TIMELESS, BHLHE40, TIPIN, SERPINE1, NPAS2, SENP3, NR1D1, and GSK3B were highly upregulated, whereas VIP, PER3, CRY2, RORB, ARNTL, VIPR2, ADCYAP1, RORA, KLF10, and PER1 were significantly suppressed in both colon cancer and rectal cancer (Figure 1(a)). In order to further demonstrate the prognostic value of CCGs in CRC, we analyzed the correlation between disease-free survival time and the expression of CCGs in CRC. Higher levels of REV1, ADCYAP1, CSNK1D, NR1D1, CSNK1E, and CRY2 had a strong link with shorter DFS time in CRC patients (Figures 1(b)–1(g)). Mutation data was retrieved and shown using the “maftools” package in R software to find CCG somatic mutations in CRC. The mutation frequency of CCGs in CRC patients was shown in a horizontal histogram, such as PER3 (5%), ARNTL2 (4%), PER1 (4%), REV1 (4%), TIMELESS (4%), ARNTL (3%), CSNK1D (3%), KLF10 (3%), and NR1D1 (3%) (Figure 1(h)). Of note, we observed that CRC patients with mutations of CCGs had a shorter DFS time (Figure 1(i)), demonstrating that CCGs have an important regulatory role in CRC development.

### 3.2. Construction and Evaluation of the Effectiveness of Prognostic Signatures

The circadian clock gene-related signature was then created by further downscaling the CCGs using Lasso regression (Figures 2(a)–2(b)). The risk score was calculated for each CRC case, risk score = (0.0184)∗ADCYAP1 + (0.2999)∗CRY2 + (0.5958)∗CSNK1D + (0.0797)∗NPAS2 + (0.1034)∗NR1D1 + (−0.0141)∗RORC. Patients were divided into low- and high-risk groups based on the median risk score of all CRC cases, and the analysis revealed a significant survival benefit for low-risk CRC patients (Figure 2(c)). KM plotter analysis demonstrated that CRC patients with a higher risk score had a shorter DFS time (Figure 2(d)) with an AUC value of 0.75, 0.71, and 0.841 for the 1-year, 3-year, and 5-year DFS, respectively (Figure 2(e)).

### 3.3. Four Prognostic CCGs Were Correlated to Immune Cell Infiltration in CRC

Figure 3(e) depicts the relationship between immune cell infiltration and expression of ADCYAP1, CRY2, NPAS2, and CSNK1D by using TIMER database. NPAS2 expression was considerably positively correlated with CD4+ T cell infiltration but dramatically negatively correlated to CD8+ T cell infiltration (Figure 4(a)). In CRC, ADCYAP1 expression was substantially associated with the levels of infiltration of CD4+ T cell, CD8+ T cell, macrophage, neutrophil, and dendritic cell (Figure 4(b)). CRY2 and CSNK1D expression was found to be substantially linked with levels of CD4+ T cell, macrophage, neutrophil, and dendritic cell infiltration in CRC (Figures 4(c) and 4(d)).

Moreover, we observed that SIGLEC15, CD274, HAVCR2, PDCD1LG2, LAG3, PDCD1, CTLA4, and TIGIT were higher in ADCYAP1 and NPAS2-high CRC samples than in ADCYAP1 and NPAS2-low CRC samples (Figures 4(e) and 4(g)). HAVCR2, TIGIT, and SIGLEC15 were higher in CRY2-high CRC samples than in CRY2-low CRC samples (Figure 4(f)). However, CD274, HAVCR2, and PDCD1LG2 were lower in CSNK1D-high CRC samples than in CSNK1D-low CRC samples (Figure 4(h)).

### 3.4. Four CRC Subtypes Were Delineated Based on the CCGs

Next, 29 circadian clock gene expressions were used to categorize the TCGA CRC data into different CRC subtypes. According to the CDF curves of the consensus score, a value of *k* = 3 was chosen to reflect stable clusters (Figures 5(a) and 5(b)). Finally, 620 CRC tumor samples were divided into 3 categories, namely, cluster1 (*n* = 428), cluster2 (*n* = 83), and cluster 3 (*n* = 109), based on the expression levels of the CCGs (Figures 5(c)–5(d)). Clusters 2 and 3 had significantly shorter overall and disease-free survival time than cluster 1 (Figures 5(e)). Cancer progression involves the progressive loss of a differentiated phenotype and the acquisition of progenitor/stem cell-like characteristics. Thus, we calculated the stemness of CRC samples in different subtypes using the logistic regression machine learning algorithm (OCLR) provided by Malta et al. based on the mRNA expression signature. The stemness score in cluster 1 and cluster 2 was considerably higher than that in the cluster 3 CRC samples (Figure 5(f)).

### 3.5. Clinical Profiles of the Four Subtypes

The distribution of gender, race, T stage, N stage, M stage, grade, and metastasis was compared across patients with the three CCG subtypes to evaluate the clinical importance of CCG-related classification. Clinically, we found that the C3 subtype had a considerably higher percentage of T3 and T4 than groups C1 or C2. In addition, we revealed that the C3 subtype had a considerably higher percentage of N1 and N2 samples than groups C1 or C2. However, the C1 subtype had a highest percentage of N0 samples than groups C2 or C3. Moreover, groups C3 had a higher percentage of grades III and IV and a lower proportion of grades I and II than cluster 1 and cluster 2. However, the distribution of gender, race, M stage, and metastasis does not have a significant difference among these clusters (Figures 3(a)–3(g)).

### 3.6. Distinct Characteristics of Immunogenicity of the CRC Subtypes

We next investigated microenvironmental variables and tumor-infiltrating lymphocyte inflation among CRC subtypes using RNA expression data. We observed that T cell CD4+ Th1, T cell NK, T cell CD4+ effector memory, T cell CD4+ central memory, and eosinophil cells were considerably enriched in cluster 2 CRC samples. Hematopoietic stem cell, endothelial cell, myeloid dendritic cell activated, M1 and M2 macrophages, monocyte, and myeloid dendritic cells were considerably enriched in cluster 3 CRC cases compared to those of clusters 1 and 2. Meanwhile, we observed that naive CD8+ T cell, common lymphoid progenitor cells, CD4+ memory T cells, CD4+ Th2 T cells, and T cell gamma delta were substantially more abundant in cluster 1 CRC samples than those of clusters 2 and 3 (Figure 6(a)).

Moreover, the expression levels of 8 immune checkpoint targets, which are critical for immunological control, were also evaluated, including SIGLEC15, CD274, HAVCR2, PDCD1LG2, LAG3, PDCD1, CTLA4, and TIGIT. As presented in Figure 7, we observed that these immune checkpoint markers in cluster 3 CRC samples were substantially higher than those in cluster 1 and 2 CRC samples (Figure 6(b)). Immune therapy was only approved for MSI-H/dMMR CRC. Thus, the destitution of MSI levels in 3 CCG subtypes was also evaluated. However, we do not observe a significant difference among 3 CCG subtypes.

### 3.7. Pancancer Analysis of CSNK1D

The present study has demonstrated the significant correlation between immune inflation and prognosis and CSNK1D in CRC. Next, we evaluated the clinical importance of CSNK1D across human cancers using the TCGA database. As presented by the forest plot, we observed that higher levels of CSNK1D were correlated to shorter DFS time in CHOL (cholangiocarcinoma), COAD (colon cancer), LIHC, and PRAD (prostate cancer); however, higher expression of CSNK1D was correlated to longer DFS time in BRCA and OV (ovarian cancer) (Figure 7(a)). By analyzing CSNK1D expression between tumor samples and normal samples, we revealed that CSNK1D was downregulated in ACC, BLCA, BRCA, CESC, COAD, DLBC, ESCA, LUAD, LUSC, PRAD, READ, STAD, TGCT, THCA, UCEC, and UCS but was increased in CHOL, GBM, HNSC, KIRP, LGG, LIHC, PAAD, and PCPG (Figure 7(b)).

Pancancer immune inflation analysis showed that CSNK1D was correlated to multiple types of immune cell inflation in various cancer types, such as LGG, COAD, KIRP, LIHC, PRAD, THCA, BLCA, BRCA, THYM, and UCEC (Figure 7(c)).

## 4. Discussion

The circadian system's significance in carcinogenesis is well recognized, and numerous studies have found differential clock gene expression in cancers compared to healthy tissues. By analyzing the TCGA database, the present study demonstrated that multiple CCGs were dysregulated and frequently mutated in CRC samples. The higher expression levels of REV1, ADCYAP1, CSNK1D, NR1D1, CSNK1E, and CRY2 had a strong link with shorter DFS time in CRC patients, demonstrating that CCGs had an important regulatory role in CRC development. ADCYAP1 is known to modulate the immune system and is involved in cell proliferation and apoptosis in normal cells [31]. ADCYAP1 upregulation or downregulation has been identified in a variety of malignancies [31]. A significant percentage of ADCYAP1 hypermethylation is frequently reported in ovarian cancer [32]. ADCYAP1 promoter hypermethylation levels have been linked to cervical cancer development [31]. The low rate of ADCYAP1 hypermethylation in early-stage lesions and its increase with the tumor stage suggest that ADCYAP1 hypermethylation may hinder ADCYAP1's apoptotic action. Cry1 expression was increased in right colon cancers but not in left colorectum tumors [33]. CRY2NK1 upregulation is associated with a worse outcome in patients with hepatocellular cancer. NPAS2 is a circadian gene that has attracted the interest of researchers due to its various effects on cells and various roles in disease development, especially cancer. Differential NPAS2 expression has been associated with patient outcomes in tumors, lung tumors, non-Hodgkin's lymphoma, and other diseases [34], and nucleotide variants in the NPAS2 gene were related to cancer patients' outcomes. In endometrial cancer of the uterus, the circadian gene NPAS2 operates as a potential tumor stimulator. NPAS2 increases liver fibrosis in hepatocellular carcinoma by direct transcriptional activation of Hes1 in hepatic stellate cells and induces glucose metabolism reprogramming and cell survival by transactivating CDC25A in liver cancer cells. Here, we constructed a prognostic signature based on CCG expression in CRC. Risk score = (0.0184)∗ADCYAP1 + (0.2999)∗CRY2 + (0.5958)∗CSNK1D + (0.0797)∗NPAS2 + (0.1034)∗NR1D1 + (−0.0141)∗RORC. KM plotter analysis demonstrated that CRC patients with a higher risk score had a shorter DFS time.

CRC is the leading cause of cancer mortality worldwide. CRC, similar with many other cancers, is a heterogeneous disease, making it a clinical challenge to enhance treatment efficacy to reduce morbidity and mortality. CRC can be caused by a number of pathogenic mechanisms, such as DNA mismatch repair failure (MMR), and epigenetic changes. A greater understanding of biology, particularly the clinical features that distinguish CRC patients, is required for more robust targeted therapy development and the application of personalized therapy. A rising corpus of research has addressed the topic of molecular categorization of CRC in recent decades in order to supplement the current staging systems, enhance therapy options, and better predict survival following treatment. The application of high-throughput sequencing has heralded a new age in subtyping research; for example, the CRC Subtyping Consortium reported the finding of four consensus molecular subtypes (CMS) in 2015, giving the most rigorous CRC classification system to date [35]. The colorectal cancer molecular classification consists mostly of mutation-centered CRC classification and transcriptome-centered CRC classification [35]. According to recent studies, intratumoral heterogeneity is best described at the transcriptome level, as it provides more comprehensive genomic information about the disorder process. The classification of CRCs based on transcriptomes has switched from supervised to unsupervised. Transcriptome-based techniques, as opposed to histopathological subtypes and traditional mutation-oriented stratification, use genome-wide expression profiling for unsupervised data processing [35]. This approach has been utilized successfully in a wide range of malignancies, including lung cancer, prostate cancer, and gastric cancers. Recent efforts have been made, like with other malignancies, to subtype CRC. Wang and colleagues, for example, used fresh-frozen tissue samples from a large multicenter cohort (CIT cohort) of 566 CRC patients to perform gene expression analysis, identifying six CRC subgroups with distinct molecular signatures and clinical correlations [35]. In this study, 513 CRC tumor samples were divided into 3 categories, namely, cluster 1 (*n* = 203), cluster 2 (*n* = 296), and cluster 3 (*n* = 296), based on the expression levels of the CCGs (Figure 2(a)). Clinical significance analysis showed that clusters 2 and 3 had significantly shorter overall and disease-free survival time than cluster 1. The stemness scores in cluster 1 and cluster 2 were significantly higher than those of cluster 3 CRC samples. Clinically, we found that the C3 subtype had a higher percentage of T3/T4, N1/N2, and grades III and IV than groups C1 or C2.

A growing body of evidence supports the importance of immune infiltration in cancer, which comprises lymphocytes, dendritic cells, and macrophages, demonstrating a wide range of patient-patient variability [36]. TILs reflect the host immune response to tumor cells, which is related to CRC patients' prognosis [37]. CD8+ cytotoxic T cells can directly destroy tumor cells. CTL is activated by type 1 helper T lymphocytes (Th1s), whereas humoral immunity is stimulated by type 2 helper T lymphocytes (Th2s). Immune responses and TILs have been studied in CRC as a strategy of classifying tumors and as prognostic indicators. TILs situated near the tumor boundary are activated and assault the tumor when PD-1 is suppressed. Most tumor-infiltrating lymphocyte types have recently been investigated, and it appears that CD8+ T cells have the greatest impact on patient outcome [38]. More than a decade ago, researchers looked into the prognostic relevance of CD8+ CTLs in a large CRC cohort. According to several studies, increased CTL levels in the tumor microenvironment have been linked to antitumor effects and improved prognosis in a variety of malignancies, including CRC. The dMMR group had more CD56+ cells, CD4+ cells, and higher CD8 protein levels than the pMMR group, according to Bai and colleagues [39]. In the present study, we observed that T cell CD4+ Th1, T cell NK, T cell CD4+ effector memory, T cell CD4+ central memory, and eosinophil cells were enriched in cluster 2 CRC samples. Hematopoietic stem cell, endothelial cell, myeloid dendritic cell activated, M1 and M2 macrophages, monocyte, and myeloid dendritic cells were considerably enriched in cluster 3 CRC cases compared to clusters 1 and 2. Meanwhile, we observed that CD8+ naive T cell, common lymphoid progenitor, and CD4+ memory/Th2 T cells were substantially more abundant in cluster 1 CRC samples than in clusters 2 and 3. Immune therapy was only approved for MSI-H/dMMR CRC. Thus, the distribution of MSI levels in 3 CCG subtypes were also evaluated. However, we do not observe a significant difference among 3 CCG subtypes. These results indicate that microsatellite-stable (mss) CRC patients may also benefit from immune therapy by using CCG-related biomarkers.

Here, we for the first time demonstrated the significant correlation between immune inflation and prognosis and CSNK1D in CRC. CK1*δ* is a member of the CK1 family. The role of CK1 has been increasingly described during the last few decades, both physiologically and pathologically. Indeed, dysregulated CK1 expression and activity have been identified in several cancers as well as neurological illnesses such as Alzheimer's disease. CSNK1D has been identified as a possible gene driver in cutaneous squamous cell cancer [40]. In patients with superficial and invasive bladder cancer, the CSNK1D gene is elevated. In bladder cancer cells, CK1 knockdown reduced catenin expression and hindered cell proliferation. Next, we evaluated the clinical importance of CSNK1D across human cancers using the TCGA database. Pancancer analysis indicates that the expression of CSNK1D was correlated to shorter DFS time in multiple cancer types, such as COAD and LIHC, and was dysregulated in various cancers, which was consistent previous reports. For example, Liu et al. reported that CSNK1D levels are strongly upregulated in HCC samples [41]. Upregulation of CSNK1D is associated with a poor prognosis for HCC patients. CSNK1D expression was higher in hepatocellular carcinoma (HCC) with distant metastasis than in HCC without metastasis [42]. According to the GSEA enrichment analysis, CSNK1D influences the HCC prognosis mostly through the cell cycle and the WNT pathway. In prostate cancer, 9 CCGs, including CSNK1D, were identified as key prognostic genes [11]. These results showed that CSNK1D may serve as an important cancer regulator.

Several limitations should also be noted in this study. First, only the TCGA database was used for the analysis of CCGs. More datasets should be analyzed and used to confirm the TCGA results. Secondly, the clinical samples would also be collected for further validation of the correlation between tumor-infiltrating lymphocytes and CCGs in the future study. Thirdly, the molecular functions of CCGs in CRC remained to be confirmed with experimental assays.

In conclusion, the present study has demonstrated that multiple CCGs were dysregulated and frequently mutated in CRC samples by analyzing the TCGA database. Higher expression levels of REV1, ADCYAP1, CSNK1D, NR1D1, CSNK1E, and CRY2 had a strong link with shorter DFS time in CRC patients, demonstrating that CCGs had an important regulatory role in CRC development. Moreover, 513 CRC tumor samples were divided into 3 categories, based on the expression levels of the CCGs. Clinical significance analysis showed that clusters 2 and 3 had significantly shorter overall and disease-free survival time than cluster 1. Stemness scores in cluster 1 and cluster 2 were significantly higher than that of cluster 3 CRC samples. Clinically, we found that the C3 subtype had a significantly higher percentage of T3/T4, N1/N2, and grades III and IV than groups C1 or C2. In addition, we reported that different CRC clusters had a significantly different tumor-infiltrating immune cell signature. Finally, pancancer analysis showed that higher expression of CSNK1D was correlated with shorter DFS time in multiple cancer types, such as COAD and LIHC, and was dysregulated in various cancers. In conclusion, we effectively developed a CCG-related predictive model and opened new avenues for research into immune regulatory mechanisms and the development of immunotherapy for CRC.

## Figures and Tables

**Figure 1:** The expression and genetic variation profile of CCGs in CRC. (a) The expression levels of CCGs in CRC and matched normal samples. (b) Correlation between disease-free survival time and expression of CCGs in CRC was present. (c) The horizontal histogram presented the genetic variation profile of CCGs in CRC. (d) CRC patients with mutations of CCGs had a shorter DFS time.

**Figure 2:** Construction and evaluation of the effectiveness of a prognostic signature. (a) LASSO coefficients for PRGs. Each curve represents a CCG. (b) 1000-fold crossvalidation of variable selection in LASSO regressions. (c) A significant survival benefit for low-risk CRC patients. (d, e) KM plotter analysis demonstrated that CRC patients with higher risk score had a shorter DFS time with an AUC value of 0.75, 0.71, and 0.841 for the 1-year, 3-year, and 5-year DFS, respectively.

**Figure 3:** Clinical profile of the four subtypes. (a–g) The distribution of gender, race, T stage, N stage, M stage, grade, and metastasis was compared across patients with the three CCG subtypes to evaluate the clinical importance of CCG-related classification.

**Figure 4:** Four prognostic CCGs were correlated to immune cell infiltration in CRC. (a–d) The relationship between immune cell infiltration and expression of NPAS2, ADCYAP1, CRY2, and CSNK1D was analyzed by using TIMER database. (e–h) The expression levels SIGLEC15, CD274, HAVCR2, PDCD1LG2, LAG3, PDCD1, CTLA4, and TIGIT were analyzed between NPAS2, ADCYAP1, CRY2, and CSNK1D-high and low groups.

**Figure 5:** Four CRC subtypes were delineated based on the CCGs. (a, b) Consensus clustering cumulative distribution function (CDF) and relative change in the area under the CDF curve (CDF delta area) were analyzed. (c) Finally, 513 CRC tumor samples were divided into 3 categories, namely, cluster 1 (*n* = 203), cluster 2 (*n* = 296), and cluster 3 (*n* = 296), based on the expression levels of the CCGs. (d) PCA analysis of 3 cluster. (d) Clusters 2 and 3 had significantly shorter overall and disease-free survival time than cluster 1. (e) The results showed that the stemness scores in cluster 1 and cluster 2 were significantly higher than those in cluster3 CRC samples.

**Figure 6:** Distinct characteristics of immunogenicity of the CRC subtypes. (a) Tumor-infiltrating lymphocyte inflation among CRC subtypes was analyzed by using RNA expression data. (b) The expression levels of 8 immune checkpoint targets, which are critical for immunological control, were also evaluated, including SIGLEC15, CD274, HAVCR2, PDCD1LG2, LAG3, PDCD1, CTLA4, and TIGIT. (c) The MSI levels in CCG-related subtypes were analyzed.

**Figure 7:** Pancancer analysis of CSNK1D. (a) Forest plot of CCGs in pan cancers. The graphic depicts the *P* value, hazard ratio, and associated 95 percent confidence interval for CCGs. (b) CSNK1D expression between tumor samples and normal samples were analyzed in pancancers. (c) Pancancer immune inflation analysis showed that CSNK1D was correlated to multiple types of immune cell inflation in various cancer types.

## Data Availability

All the data can be acquired by reasonable request.
